The article "Painting Classification in Art Teaching under Machine Learning from the Perspective of Emotional Semantic Analysis" was retracted in 2023. Reasons: unreliable results or conclusions; concerns about the data; concerns about the results or conclusions; concerns about the peer review.

# Painting Classification in Art Teaching under Machine Learning from the Perspective of Emotional Semantic Analysis

**DOI:** 10.1155/2022/9592050

**Published:** 2022-05-02

**Authors:** Jia Liang, Zhenqiu Xiao

**Affiliations:** ^1^Lin Fengmian Academy of Fine Arts, Jiaying University, Meizhou 514015, Guangdong, China; ^2^School of Computer, Jiaying University, Meizhou 514015, Guangdong, China

## Abstract

This paper aims to explore the Painting Classification in art teaching under Machine Learning. Based on Emotional Semantics and Machine Learning, the Emotional Semantics of the traditional image are expounded. Firstly, Emotional Semantics are applied to figure painting in art teaching. Then, the convolutional sparse automatic encoder model is introduced in Painting Classification. Finally, the accuracies of the Painting Classification of the Support Vector Machine classifier (SVMC) and that of the Naive Bayes classifier are compared, and the relevant conclusions are drawn. The accuracy of Painting Classification is positively correlated with the scale of painting. After analysis, the painting set is classified in a ratio of 2 : 1, with 2/3 as training set and 1/3 as test set, which is conducive to the good accuracy of classification. In Machine Learning, proper whitening can improve the accuracy of Painting Classification to a certain extent. However, when the whitening treatment coefficient is selected, it cannot be too large, and the average pooling is more accurate than maximum pooling. After the comparison of the new SVMC, the Naive Bayes classifier, and the convolutional sparse automatic encoder, the convolutional sparse automatic encoder has the highest accuracy of Painting Classification. Therefore, the Painting Classification in art teaching under Machine Learning is explored, which is of great help to the classification work of students or teachers in the future.

## 1. Introduction

With the rapid development and application of computer technology, network technology, and database technology, painting has become an important carrier of information exchange [1]. Nevertheless, the teacher not only has to perform the daily teaching work but also has to organize the order classification of paintings. Consequently, how to accurately classify the paintings in art teaching has become one of the common concerns of universities. According to the different types, the paintings can be classified into ink and wash painting, oil painting, Mogu painting, Gouache painting, print, wall painting, watercolor painting, claborate-style painting, free sketch painting, and abstract painting. The figure painting, architecture painting, and landscape painting that are common in daily life are selected as the research objects. Figure painting refers to the painting of the character image as the main body, which strives to depict the character's personality vividly. Its vivid method often puts the performance of the character in the environment, atmosphere, figure, and dynamic rendering. Hence, Chinese painting theory also calls the figure painting “Chuan Shen.” Architectural painting is similar to the sketch of architects. It is a painting that just expresses architecture, but it is not the other paintings. An expressive architectural painting is an art that evokes the design intention and space. Landscape painting refers to the painting with the landscape as the theme, such as Chinese landscape painting [2].

Mandalorian [3] proposed an improved Fisher coding method, which achieved better classification results for fine art painting images with less training data. Saussure [4] proposed a local feature called Classemes based on natural images and verified that the local features of Classemes can make the image content more natural. Kahn [5] put forward a new extraction method by exploiting an ensemble of edge detections and applying the texture patterns based on these extracted edges to distinguish the Van Gogh from non-Van Gogh works. These two existing works fully consider the brushstroke information in art painting images and achieve good results in the classification task of art painting images. However, the datasets they use are very limited in size, and the models are only built for two-class classifications. Azizan et al. [6] compared the classification methods of nearest neighbor and Support Vector Machine (SVM) on the classification task of art painting images and found that the classification performance of the nearest neighbor classifier was better than that of the Support Vector Machine classifier (SVMC). Nelloh [7] proposed an end-to-end idea to integrate the extraction, processing, and classification of image features to help deep mining and extraction of image information. From the perspective of the processing of the AlexNet convolutional layer, the feature map obtained by the shallow convolution is the image edge, color, and other shallow features, and the feature maps obtained by deep convolution are the abstract features of the overall outline of the image, which are the deep features.

In this context, the accuracy of Painting Classification in art teaching is analyzed under Machine Learning starting from Emotional Semantics. Firstly, Emotional Semantics are applied to the Painting Classification in art teaching, and then the convolution sparse automatic encoder in Machine Learning is applied. The Painting Classification accuracies of the SVMC, the Naive Bayes classifier, and the convolutional sparse automatic encoder are compared for the accuracy of the experimental data. The objective of this work is to provide a methodological reference for analyzing the accuracy of Painting Classification in art teaching.

## 2. Methods

### 2.1. Traditional Image Emotional Semantics

The traditional image emotional semantic analysis principle under Machine Learning is as follows. Firstly, an appropriate emotional space representation model is selected, and the visual features are extracted such as color and texture from the image content. Then, Machine Learning and color coding are used. Finally, learning and training are implemented based on the manually labeled samples, thus obtaining the image emotional detector [8].  Figure 1 shows the analytical framework.

Next, the traditional image emotion semantic analysis is discussed and summarized from three aspects: emotion model, visual feature, and Machine Learning model.

#### 2.1.1. Emotion Model

The analysis of traditional image Emotional Semantics mainly uses the general emotional model in psychology. These emotional space representation models can be classified into the Categorical Emotion States (CES) model and the Dimensional Emotion Space (DES) model [9]. The emotion representation method of the CES model is used to classify emotion into different subclasses based on the categorical concept, including hatred, sadness, desire, surprise, love, and joy. However, the emotion modelers who adopt the DES model consider that emotions not only have bipolar features but also can be decomposed into different components, and the emotions are represented with the help of Cartesian coordinates [10, 11].

#### 2.1.2. Visual Feature

Extraction of visual features is an important research content of traditional image emotional semantic analysis, which refers to using computer technology to extract feature data from image content to characterize it [12]. Different from other research topics in computer vision, the research of image emotion semantics needs to analyze the information closely related to psychology, emotion, and feeling, so it is necessary to combine human psychological and physiological features for visual feature design and representation [13]. Colors are enabled of awakening human emotions. For example, red makes people feel warm and uplifting, green makes people feel calm and comfortable, white makes people feel clean and bright, and black makes people feel solemn and sad. The texture is also a commonly used underlying visual feature, which reflects the regular organization and arrangement of the surface of an object. Although the ability of texture information to trigger emotion is not as strong as that of color, different texture structures can also trigger different emotional responses [14]. The shape is an area surrounded by closed contours, and shape features can express emotional meanings because different shapes can trigger different emotional responses [15].

#### 2.1.3. Machine Learning Model

The final task of traditional image emotion semantic analysis is to establish a reliable mapping between visual features and Emotional Semantics. Because the relationship between image features and emotion is complex, it is difficult to establish effective mapping rules completely relying on prior knowledge [16]. Machine Learning can simulate the human learning process and is an important means to achieve image emotion understanding across the semantic gap [17].

### 2.2. Machine Learning Model

Machine Learning is a science of Artificial Intelligence (AI). The main research object of this field is AI, especially how to improve the performance of specific algorithms in experiential learning. Besides, the research directions of Machine Learning mainly include Decision Tree, Random Forest, artificial neural networks, and Bayesian Learning [18].

In recent years, many methods of Machine Learning have been proposed. The classification is based on the learning strategies (Figure 2).

The common algorithms of Machine Learning are as follows.

#### 2.2.1. Decision Tree Algorithm

Decision Tree and its variants are a class of algorithms that divide the input space into different regions, with algorithms of independent parameters for each region. The Decision Tree algorithm makes full use of the tree model. The root node to a leaf node is a classification path rule, and each leaf node represents a judgment category. The sample is firstly classified into different subsets, and then they are segmented recursively until samples of the same type are obtained in each subset. The test is performed from the root node to the subtree and the leaf node, and the prediction category can be obtained [19]. This method is characterized by simple structure and high efficiency of data processing. There are three universal algorithms for the generation of the Decision Tree, among which the calculation method of information entropy is shown as follows:

(1) $$\begin{array}{c} H\left(X\right)=-\sum_{i=1}^{n}P\left(x_{i}\right)\log\;P\left(x_{i}\right). \end{array}$$

In (1), *H*(*X*) expresses the information entropy, *P*(*x*_*i*_) expresses the proportion of the classification types,  *n* expresses the number of classifications, and *i* expresses the *i*-th class. Equation (2) shows how the conditional entropy is calculated.

(2) $$\begin{array}{c} H\left(X|Y\right)=\sum_{i=1}^{n}P\left(y_{i}\right)H\left(X=x_{i}|Y\right). \end{array}$$

In (2), *H*(*X|Y*) is the conditional entropy that represents the information entropy of a single feature, and *P*(*y*_*i*_) is the proportion of some feature within its features. The meanings of the remaining letters are the same as (1). According to (1) and (2), (3) can be obtained, which shows the calculation method of information gain.

(3) $$\begin{array}{c} I\left(X,Y\right)=H\left(X\right)-H\left(X|Y\right). \end{array}$$

According to (3), information gain refers to the difference between information entropy and conditional entropy.

#### 2.2.2. Naive Bayes Algorithm

The Naive Bayes algorithm is one of the representative algorithms of Machine Learning. It is not a single algorithm but a series of algorithms, all of which share the common principle that each feature being classified is independent of the value of any other feature. Naive Bayes algorithm can help Machine Learning to achieve ideal prediction results. In the Naive Bayes classifier, each of these “features” contributes the probability independently, regardless of any correlation among features. However, these features are not always independent, so it is generally regarded as a disadvantage of the Naive Bayes algorithm [20]. In short, the Naive Bayes algorithm allows predicting a class by using the probability to give a set of features. Compared with other classification methods, the Naive Bayes algorithm requires less training. The only work that needs to be completed before the prediction is to find the parameters of the individual probability distribution of the feature, which can usually be finished quickly and precisely. This means that the Naive Bayes classifier can perform well even for the high-dimensional data points or large numbers of data points. Equation (4) shows the specific calculation.

(4) $$\begin{array}{c} P\left(A|B\right)=\frac{P\left(AB\right)}{P\left(B\right)}. \end{array}$$

In (4), *P* represents the probability. If *A* represents the white stone, *B* represents the black one. *P*(*A*∣*B*) represents the probability of picking the white stone under the conditions that the stones are from bucket B. *P*(*AB*) represents the probability of picking the white stone from bucket B, and *P*(*B*) represents that of picking the black stone.

#### 2.2.3. SVMC Algorithm

The basic idea can be summarized as follows. The space is enhanced by a nonlinear transformation. Then, the optimal linearly classified surface is obtained in the new complex space. The classification function obtained in this way is similar to the neural network algorithm in form. SVM is a representative algorithm in the statistical learning field. However, it is very different from the traditional way of thinking, and it is inputting space and improving the dimension to simplify the problem so that the problem can be reduced to a linear separable classical solution [21]. SVM is applied to spam recognition and face recognition. Equation (5) shows the specific calculation.

(5) $$\begin{array}{c} w^{T}x+b=0. \end{array}$$

In (5), *w* expresses the normal vector that determines the direction of the hyperplane, and *b* expresses the offset term that determines the distance between the hyperplane and the origin.  *x* expresses any point, and *T* expresses the hyperplane. Partition hyperplane can be denoted as (*w*^*T*^, *b*), and the distance from any point *x* to the hyperplane in the sample space can be written as

(6) $$\begin{array}{c} r=\frac{\left|w^{T}x+b\right|}{\left\|w\right\|}. \end{array}$$

In (6), *r* is the distance, and the rest of the letters have the same meanings as the above equations.

Moreover, SVM and Naive Bayes algorithms are both important algorithms in classification. The Naive Bayes algorithm is less sensitive to data due to the number of parameters estimated. SVM can solve the problems of Machine Learning under small samples. It is sensitive to real data, but its memory consumption is large, and the operating steps are also cumbersome. Consequently, both methods have advantages and disadvantages.

#### 2.2.4. Random Forest Algorithm

There are many ways to control the generation of the data tree. According to previous experience, splitting attributes and pruning are mostly preferred, but they cannot solve all the problems. Occasionally, there are some problems such as noise or excessive splitting attributes. Based on this situation, the estimation error of relevant data can be obtained by summarizing the results, which can be combined with the estimation error of test samples to evaluate the fitting and prediction accuracy of the combination-tree learner [22]. This method helps to generate high precision classifiers, deal with a large number of variables, and balance the errors among the classification datasets.

#### 2.2.5. Artificial Neural Network Algorithm

The artificial neural network is similar to the extremely complex networks of neurons, in which individual units are interconnected. Each unit has numerical inputs and outputs, and the form can be real numbers or linear combinatorial functions. It needs to learn with a learning criterion before it works. When the network is wrong, it is less likely to make the same mistake through learning. This method has strong generalization ability and nonlinear mapping ability, which can model the system with little information. From the perspective of functional simulation, it has parallelism and an extremely fast speed of information transmission [23]. Equation (7) shows its calculation.

(7) $$\begin{array}{c} Q_{a+1}=Q_{a}-c_{a}d_{a}. \end{array}$$

In (7), *Q*_*a*+1_ represents the weight and deviation values of the neuron layer, *Q*_*a*_ represents the weight and deviation values after the iterative calculation, *c*_*a*_ represents the speed of neural network learning, and *d*_*a*_ represents the gradient of the error function.

In addition, there is the specific calculation method of the space size of the convolution kernel after the cavity which is shown as follows:

(8) $$\begin{array}{c} A=\left(n-1\right)*b+1. \end{array}$$

In (8), *A* expresses the size of the convolution kernel, *n* expresses the actual size of the original convolution kernel, and *b* expresses the voidage. Equation (9) shows the specific calculation method of image size after convolution.

(9) $$\begin{array}{c} B=\frac{\left(l-K+2P\right)}{S+1}. \end{array}$$

In (9), *B* is the size of the image after convolution,  *l* is the actual input of the size of the image, *K* is the output of the size of the image, *P* is the size of the filling image, and *S* is the step size.

Deep Learning is a new research direction in Machine Learning. Machine Learning is a technology that explores how the computer simulates or realizes the learning behavior of animals to learn new knowledge or skills, rewrite the existing data structure, and improve the program performance [24]. Deep Learning is strongly related to the “neural network” in Machine Learning, which is also its main algorithm and means. Deep Learning is also the “improved neural network” algorithm [25], and Figure 3 shows its theoretical model.

Nonnegative matrix factorization (NMF) is also an effective Deep Learning method. It makes the final product approximate to the original matrix as much as possible by finding two or more nonnegative matrices, realizing nonlinear dimensionality reduction of data [26]. The calculation method of the norm cost function based on the matrix difference is shown as follows:

(10) $$\begin{array}{c} \underset{P,W,Q}{\min}{\left\|Y-\mathrm{PW}Q^{T}\right\|}_{F}^{2}. \end{array}$$

In (10), *Q*^*T*^ represents the transpose of matrix *Q*, and ‖.‖_*F*_ represents the norm of the matrix difference. *P*, *W*, *Q*, and *Y* represent different matrices. The updated decomposition calculation method is shown as follows:

(11) $$\begin{array}{c} P_{ij}⟵P_{ij}\frac{\left(YQW^{T}\right)}{{\left(PWQ^{T}QW^{T}\right)}_{ij}}. \end{array}$$

(12) $$\begin{array}{c} W_{ij}⟵W_{ij}\frac{{\left(P^{T}YQ\right)}_{ij}}{{\left(P^{T}PWQ^{T}Q\right)}_{ij}}. \end{array}$$

(13) $$\begin{array}{c} Q_{ij}⟵Q_{ij}\frac{{\left(YPW\right)}_{ij}}{{\left(QW^{T}P^{T}PW\right)}_{ij}}. \end{array}$$

In equations (11)–(13), *P*_*ij*_ represents the element in the *i*-th row and the *j*-th column of matrix *P*, *W*_*ij*_ represents the element of the *i*-th row and the *j*-th column of matrix *W*, and *Q*_*ij*_ represents the element in the *i*-th row and *j*-th column of matrix *Q*. In addition, *P*, *W*, *Q*, and *Y* represent different matrices. *W*^*T*^, *Q*^*T*^, and *P*^*T*^ represent the transpose of different matrices.

Multitask learning (MTL) is an important part of Deep Learning methods. Its principle is to solve the data fragmentation of Deep Learning by finding useful information from relevant data [27]. According to the definition of the MTL model, the specific calculation method is shown as follows:

(14) $$\begin{array}{c} \min\sum_{m}^{M}L\left(X^{m},Y^{m},W^{m}\right)+\lambda Reg\left(W\right)\;. \end{array}$$

In (14), *X*^*m*^, *Y*^*m*^, and *W*^*m*^ represent matrices *X*, *Y*, and *W* inputted by the *m*-th task, respectively; *M* represents the total number of samples; *Reg* refers to the regularization constraint, and *λ* represents the weight that controls the regularization constraints.

To ensure the accuracy of the research data, it is necessary to calculate the correct rate and recall rate, as shown in the two following equations:

(15) $$\begin{array}{c} \text{Accuracy}=\frac{TP+TN}{P+N}. \end{array}$$

(16) $$\begin{array}{c} \text{Recall}=\frac{TP}{TP+FN}=\frac{TP}{P}. \end{array}$$

In (15) and (16), *TP* represents the number of correctly divided positive examples, *TN* represents the number of correctly divided negative examples, *P* represents TP + FN, *FN* represents the number of incorrectly divided negative examples, and *N* represents the total number.

The convolutional neural network (CNN) model includes convolutional calculations and feedforward neural networks with deep structures. It is mainly divided into four parts: input layer, convolutional layer, pooling layer, and fully connected layer. It is one of the representative algorithms under Deep Learning [28].

Equations (17)–(21) show the specific calculation method.

(17) $$\begin{array}{c} R_{t}=ℑ\left(B_{t}\left[b_{t-1},x_{t}\right]+P_{f}\right). \end{array}$$

(18) $$\begin{array}{c} Y_{t}=ℑ\left(A_{I}\cdot \left[b_{t-1},x_{t}\right]+P_{I}\right). \end{array}$$

(19) $$\begin{array}{c} Z_{t}=\tan\;b\left(B_{D}\cdot \left[b_{t-1},x_{t}\right]+C_{D}\right). \end{array}$$

(20) $$\begin{array}{c} D_{t}=T_{t}\times D_{t-1}+I_{t}\times D_{t}. \end{array}$$

(21) $$\begin{array}{c} E_{t}=\partial \left(A_{E}\left[b_{t-1},x_{t}\right]+C_{E}\right). \end{array}$$

In equations (17)–(21), *R*_*t*_, *Y*_*t*_, and *E*_*t*_ represent the forget gate, input gate, and output gate, respectively; ℑ represents the hidden layer neuron; *B*_*t*_ represents the model output; *b*_*t*−1_ represents the hidden layer information at the *t* − 1 time; *x*_*t*_ represents the input at time *t*; *P*_*f*_ and *P*_*I*_ represent the activation functions of the forget gate and the input gate, respectively; *Z*_*t*_ refers to the candidate memory cell information; *b* is the function coefficient; *B*_*D*_ represents the bias of the convolution kernel; *C*_*D*_ and *T*_*t*_ represent the maximization pool and average pooling, respectively; *D*_*t*−1_ stands for the hidden layer of candidate memory information, *A*_*E*_ represents the probability obtained by the function, and *C*_*E*_ is the word vector dimension.

When the automatic encoder is applied to the field of image and vision, if the image size is relatively small, the whole image can be stored in vector form, and feature learning and training can be performed. Nevertheless, in the case of large image size, this method requires too much computation and is not easy to be implemented. Therefore, for large-size images, instead of processing the whole image directly, the convolutional automatic encoder model is adopted to learn the local features in small image blocks. Subsequently, the global features of the image are extracted with the help of the convolutional network according to the stationary features of the image. The overall scheme is adopted in image classification based on the convolutional sparse automatic encoder (Figure 4).

The image classification system of convolutional sparse automatic encoder consists of the local feature learning based on sparse automatic encoder, global feature extraction based on convolutional network, and image classifier. Such a classification system is helpful to solve the problem of accurate image classification from all levels. The convolutional sparse automatic encoder is mainly responsible for the local image recognition by using whitening processing and principal component analysis. In Machine Learning, the convolution operation in the convolutional network is adopted to scan the image, and the local feature weight is used as the detector to obtain the global feature response. When the data is good, it is classified in the image classifier.

### 2.3. Key Technologies to be Adopted

The first is whitening processing: The training data is assumed to be an image, and the input is redundant when used for training due to the strong correlation between adjacent pixels in the image. The purpose of whitening is to reduce the redundancy of the input. It means that through the whitening process, the input of the learning algorithm has the following properties. Firstly, the correlation between features is low. Then, all features have the same variance. The second is principal component analysis method: Many original indicators with certain correlations (such as *P* indicators) are combined into a new set of independent comprehensive indicators to replace the original indicators. The third is case study method: Through the collection of relevant data, it can find out the process of Painting Classification and analysis in art teaching based on Machine Learning from the perspective of emotional semantic analysis by experts and scholars, thus establishing a corresponding research framework and making the article more scientific. The fourth is comparative analysis method: It refers to the multiway comparison of two or more research objects to discover the similarities and differences between them and to analyze and learn from good methods. The purpose is to provide a good strategy for Painting Classification in art teaching. The fifth is quantitative and qualitative analysis method: It refers to a common method of analyzing, researching, and summarizing the features of quantities, the logical relationship among quantities, and the changing trend of quantities by collecting relevant research data. The qualitative analysis method refers to the method in which forecasters analyze the future development trend and nature of the data according to relevant historical data changes, government policy announcements, and major social events with influence.

## 3. Results

### 3.1. Application of Emotional Semantics in Painting Classification in Art Teaching

To analyze the classification of painting in art teaching, the painting works of students of a fine arts college are selected as the research objects, and the convolutional sparse automatic encoder is adopted for image classification. Due to a large number of categories, the figures, buildings, and landscapes are selected only.  Figure 5 shows the specific results.

Table 1 shows the concrete numerical results.

As given in Figure 5, the accuracy of Painting Classification is closely correlated to the number of drawings. As the size of the drawing set decreases, the accuracy of the classification also decreases. The larger the proportion of the drawing set is, the higher the accuracy of the classification is. When the size of the drawing set is less than half of the total, the classification accuracy slowly decreases, but the gap between the two will not be large. Therefore, the larger the plot set size is, the higher the final classification accuracy is.

4/5 of the drawing set are selected as the training set and 1/5 are included in the test set to discuss the impact of Emotional Semantics on different drawing types. The specific results are shown in Figure 6.

Table 2 shows the concrete numerical results.

In Figure 6, the smaller the selected painting training set, the lower the final image classification accuracy. However, the larger the selected painting training set is, the higher the image classification accuracy is, and there is a slight decrease after increasing to the peak value. Conversely, it is generally difficult to obtain higher accuracy with a smaller training set, but it is not the case that the larger the training set, the better. After the verification of the above two experiments, the painting set can be divided into a ratio of 2 : 1, of which 2/3 is used as the training set and 1/3 is used as the test set. Such a division standard is conducive to obtaining better classification performance.

### 3.2. Application of Machine Learning in Painting Classification in Art Teaching

The CNN model in Machine Learning is applied to analyze the accuracy of Painting Classification.  Figure 7 shows the specific results.

Table 3 shows the concrete numerical results.

In the pooling layer area of 15 ∗ 15, the classification accuracy of the drawing is 75.44, 74.53, 81.31, and 80 when whitening coefficient is 0, 1, 0.1, and 0.01, respectively; in max pooling, the classification accuracy is 77.75, 74.97, 79.84, and 77.5 when the whitening coefficient is 0, 1 0.1, and 0.01, respectively. In the pooling layer area of 5 ∗ 5, the classification accuracy is 72.53, 73.53, 78.38, and 75.97 when the whitening coefficient is 0, 1, 0.1, and 0.01, respectively; in max pooling, the classification accuracy of the drawing is 75.34, 74.25, 77.56, and 74.56 when the whitening coefficient is 0, 1, 0.1, and 0.01, respectively. From these data, it can be found that, no matter what parameters are used, proper whitening can improve the accuracy of Painting Classification to a certain extent. However, when the whitening processing coefficient is determined, it should not be too large. From the data in the figure, it can be found that when the coefficient is 1, the final accuracy rate of nonwhitening is not high.

In addition, an overlapping pooling method is now used to explore the image classification accuracy under different whitening conditions.  Figure 8 shows the specific results.

Table 4 shows the concrete numerical results.

Figure 8 illustrates that when the pooling area is determined and the pooling step size is 10, the accuracy is 75.8 without whitening and is 81.34 with whitening under average pooling; the accuracy is 78.12 without whitening and 80.22 with whitening under the max pooling. When the step size is 5, the accuracy is 76.06 without whitening and 81.78 with whitening under average pooling; and the accuracy is 78.56 without whitening and 80.5 with whitening under max pooling. From these data, it can be found that the whitening process greatly improves the accuracy of the Painting Classification, and the accuracy under max pooling is higher compared with the value under average pooling.

### 3.3. Plot Categorical Data Results under Different Classifiers

To more accurately analyze the effect of Machine Learning on Painting Classification in art teaching, two different classifiers are introduced for comparison, which are Naive Bayes classifier and SVMC.  Figure 9 shows the specific results.

Table 5 shows the specific numerical results.

In Figure 9, the accuracy of the SVM classifier is 86.1% for figure painting, 86.5% for architecture painting, and 90% for landscape painting. The accuracy of the Naive Bayes classifier for figure, architecture, and landscape paintings is 84.5%, 84.5%, and 82.1%, respectively. The accuracy of the convolutional sparse automatic encoder for figure, architecture, and landscape paintings is 80%, 95%, and 92.8%, respectively. It indicates that the accuracy of the SVM classifier is relatively stable, with the highest accuracy in the landscape painting; the Naive Bayes has the lowest accuracy of Painting Classification, while the convolutional sparse automatic encoder has the highest accuracy of Painting Classification. The convolutional sparse automatic encoder achieves the highest accuracy in the Painting Classification of architecture painting. It is possibly related to the features of architectural images themselves, which are easier to be identified than the other two kinds of images. Furthermore, in the task of natural image classification based on Machine Learning, the quite typical method is the natural image classification based on the word bag model. The word bag model is derived from the field of natural language processing. The main idea is understanding the natural image as a sentence and representing its features with a bag composed of words that can be words and phrases in the sentence. The framework of the word bag model mainly includes feature extraction, feature coding, and classifier design. Compared with the Painting Classification of Emotional Semantics mentioned in this work, the feature extraction in the word bag model is the most critical step, but this process not only consumes time but also requires much manpower and material resource. Therefore, the Emotional Semantics analysis is superior.

## 4. Conclusion

Painting Classification in art teaching is a task that both teachers and students need to complete. From the perspective of Emotional Semantics analysis, the Machine Learning algorithm is adopted to investigate the Painting Classification in art teaching. There are several conclusions. The accuracy of Painting Classification is related to the number of paintings. The smaller the scale of painting is, the lower the accuracy is; and the larger the scale is, the higher the accuracy is. The painting set is classified in the ratio of 2 : 1, with 2/3 as the training set and 1/3 as the test set. Such classification standard is conducive to good classification performance. Proper whitening can improve the accuracy of Painting Classification to a certain extent. The classification effects of the introduced SVM, Naive Bayes, and convolutional sparse automatic encoder are compared. The results reflect that the average accuracy of the convolutional sparse automatic encoder is 89.27%, that of SVM is 87.53%, and that of Naive Bayes is 84.36%. The accuracy of the convolutional sparse automatic encoder is the highest. Due to the limited energy, this work has some limitations in data acquisition, which leads to some deviations in the analysis of relevant data. In addition, from the perspective of Emotional Semantics analysis, the economic input of Painting Classification under Machine Learning in art teaching is not discussed, and the benefit evaluation can be performed according to the specific situation. Furthermore, in the future, various types of art painting can be considered, such as Chinese landscape painting, ink and water painting, and western oil painting, so that Machine Learning can optimize and improve the accuracy of Painting Classification.

## Figures and Tables

**Figure 1:** Framework for traditional image emotional semantic analysis.

**Figure 2:** Classification of Machine Learning.

**Figure 3:** Deep Learning model.

**Figure 4:** Image classification and processing system under convolutional sparse automatic encoder.

**Figure 5:** The impact of Emotional Semantics on different types of paintings (Figure (a): the impact when the training set ratio is greater than or equal to 0.5; Figure (b): the impact when the training set ratio is less than 0.5).

**Figure 6:** The impacts of Emotional Semantics on different types of paintings when the training set is selected (Figure (a): the results when the proportion of the training set is less than or equal to 0.5; Figure (b): the results when the proportion of the training set is greater than 0.5).

**Figure 7:** Image classification accuracy under different pooling conditions (Figure (a): the results when the pooling area is 15 ∗ 15; Figure (b): the results when the pooling area is 5 ∗ 5).

**Figure 8:** Image Painting Classification accuracy in overlapping mode.

**Figure 9:** Comparison of classification performances of three classifiers.

**Table 1:** The effect of Emotional Semantics on different types of painting.

Training set proportion	Training set proportion	Character class	Architecture	Landscape
<0.5	1/3	0.799	0.852	0.922
	1/4	0.784	0.853	0.918
	1/5	0.782	0.849	0.917

≥0.5	4/5	0.811	0.882	0.942
	3/4	0.804	0.871	0.938
	2/3	0.82	0.86	0.932
	1/2	0.806	0.859	0.923

**Table 2:** The effect of Emotional Semantics on different types of painting when selecting training sets.

Training set proportion	Training set proportion	Character class	Architecture	Landscape
≤0.5	0.1	0.752	0.794	0.884
	0.2	0.754	0.805	0.915
	0.3	0.779	0.807	0.917
	0.4	0.785	0.837	0.928
	0.5	0.798	0.859	0.925

>0.5	0.6	0.801	0.826	0.913
	0.7	0.816	0.866	0.921
	0.8	0.83	0.88	0.932
	0.9	0.826	0.878	0.932
	1	0.818	0.861	0.927

**Table 3:** Accuracy of image classification under different pooling conditions.

Pool area	Pooling method	Nonwhitening	Whitening coefficient 1	Whitening coefficient 0.1	Whitening coefficient 0.01
15 ∗ 15	Average pooling	75.44	74.53	81.31	80
	Maximum pooling	77.75	74.97	79.84	77.5

5 ∗ 5	Average pooling	72.53	73.53	78.38	75.97
	Maximum pooling	75.34	74.25	77.56	74.56

**Table 4:** Accuracy of image Painting Classification in the overlapping mode.

Pooling method	Nonwhitening	Whitening
Average pooling (step 10)	75.8	81.34
Maximum pooling (step 10)	78.12	80.22
Average pooling (step 5)	76.06	81.78
Maximum pooling (step 5)	78.56	80.5

**Table 5:** Comparison of classification performances of three classifiers.

Type	Support vector machine	Naive Bayes	Convolutional sparse automatic encoder
Character class	86.1	84.5	80
Architecture	86.5	84.5	95
Landscape	90	82.1	92.8

## Data Availability

The data used to support the findings of this study are included within the article.
